# Optimizing heat source distribution in sintering molds: Integrating response surface model with sequential quadratic programming

**DOI:** 10.1016/j.heliyon.2024.e29376

**Published:** 2024-04-09

**Authors:** Sanli Liu, Min Chen, Nan Zhu, Zhouyi Xiang, Songhua Huang, Shunqi Zhang

**Affiliations:** a School of Advanced Technology, Xi'an Jiaotong-Liverpool University, Suzhou, China; b ZINSIGHT Technology (Shanghai) Co., Ltd, Shanghai, China; c School of Mechatronic Engineering and Automation, Shanghai University, Shanghai, China

**Keywords:** Temperature uniformity, Sintering mold, Response surface methodology, Sequential quadratic programming, Optimal design

## Abstract

The sintering mold imposes strict requirements for temperature uniformity. The mold geometric parameters and the power configuration of heating elements exert substantial influence. In this paper, we introduce an optimization approach that combines response surface models with the sequential quadratic programming algorithm to optimize the geometric parameters and heating power configuration of a heating system for sintering mold. The response surface models of the maximum temperature difference, maximum temperature, and minimum temperature of the sintering area are constructed utilizing the central composite design method. The model's reliability is rigorously confirmed through variance analysis, residual analysis, and generalization capability validation. The models demonstrate remarkable predictive accuracy within the design space. A nonlinear constrained optimization model is established based on the response surface models, and the optimal parameters are obtained after 9 iterations using the sequential quadratic programming algorithm. Under the optimal parameters, the maximum temperature difference is maintained at less than 5 °C, confirming exceptional temperature uniformity. We conduct parameter analysis based on standardized effects to determine the main influencing factors of temperature uniformity, revealing that the distance between adjacent heating rods and the power density of the inner heating rods exert significant influence. Enhanced temperature uniformity can be achieved by adopting a larger distance between heating rods and configuring the power density of the heating rods to a relatively modest level. This work introduces a practical approach to optimize the heating systems for sintering molds, with potential applications in various industrial mold optimization.

**Table:** Abbreviations

ANN	Artificial neural network
ANOVA	Analysis of variance
CCD	Central composite design
FEM	Finite element method
GA	Genetic algorithm
NSGA-II	Non-dominated sorting genetic algorithm-II
PSO	Particle swarm optimization
RSM	Response surface methodology
RHCM	Rapid heat cycle molding
SQP	Sequential quadratic programming

## 1 Introduction

Silicon carbide (SiC) offers excellent electric and thermal capabilities compared to silicon. SiC power modules have been widely used in wind turbines, traction systems of electric rail vehicles, and hybrid electric vehicles, which place higher reliability requirements [1]. The strength and stability of die-attach joints significantly impact the reliability of power modules. Compared to traditional solder materials, the sintered nano-Ag exhibits robust thermal stability at temperatures exceeding 300 °C, making them an ideal high-strength die-attach material for SiC power modules [2,3]. In industrial production, the sintering process of nano-Ag paste is usually conducted within the sintering mold. The uniformity of sintering temperature significantly influences the microporous structure and electrical performance of sintered joints [[4], [5], [6]]. Therefore, ensuring temperature uniformity in the sintering area becomes crucial for enhancing the reliability of the SiC power modules.

Significant efforts have been dedicated to achieving uniform mold heating through simulation-based optimization in recent years. The optimization primarily falls into two prominent categories: optimization based on surrogate models and optimization based on physical models. The surrogate model-based optimization couples the optimization algorithms with surrogate models to ascertain optimal design parameters, offering the benefits of the simple model and high efficiency. Various surrogate models, such as response surface methodology (RSM) models [7,8] artificial neural network model (ANN) [9], and Kriging model [10], have been employed to depict the relationship between design parameters and objective function. On the other hand, the physical model-based optimization integrates the optimization algorithms with finite element models, eliminating the approximation errors inherent in surrogate models. This approach significantly enhances precision, offering a substantial advantage in applications demanding high accuracy.

Numerous studies have successfully attained enhanced temperature uniformity by optimizing the structural design of mold heating systems. Kuo et al. [11] presented a conformal heating channel to enhance the temperature uniformity of the mold surface in the LSR injection molding. Baris et al. [12] design a plastic injection mold with conformal cooling channels by metal additive manufacturing and achieved up to 62.9 % better cooling performance with a better thermal uniformity on the mold surface. Nguyen et al. [13] used the response surface methodology to design a conformal channel which provide more efficient mold heating and temperature uniform than a straight cooling channel. Li et al. [14] optimized the layout of heating rods to improve temperature uniformity by coupling the RSM model with a genetic algorithm (GA) for rapid heat cycle molding (RHCM) mold. Wang et al. [15,16] integrated particle swarm optimization (PSO) and the non-dominated sorting genetic algorithm-II (NSGA-II), respectively, with RSM models to explore the optimal geometric parameters for a heating system of RHCM mold. Xiao et al. [17] combined PSO with finite element method (FEM) to design the positions of heating rods in the RHCM mold. However, these studies have generally ignored the heating rods' power density, which substantially influences temperature uniformity. This factor becomes particularly critical in molds with constrained dimensions, where achieving desired temperature uniformity might not be feasible through geometric parameters optimization alone. Xiao et al. [18] and Li et al. [9] employed RSM-NSGA-II and ANN-NSGA-II methods to search for optimal geometric parameters and the power density of heating rods to balance the heating time and temperature uniformity. A limitation in these studies is the consistent power density setting across all heating rods. While this approach is advantageous for enhancing heating efficiency, the uniform power density setting fails to address the varying thermal demands across different areas of the mold. Therefore, more specific power density arrangements are required to improve temperature uniformity. Hao et al. [7] optimized the power of four heating rods in an injection mold by the RSM model, and the temperature uniformity was improved notably by 79 %. Xiao et al. [19] combined the sequential quadratic programming (SQP) algorithm with FEM to design the positions and power of seven heating rods in the RHCM mold. The proposed SQP-FEM methods effectively obtained the optimal design parameters compared to the simulation-based trial and error method. These investigations have focused on optimizing the power settings of heating rods in mold heating systems, assigning different power densities to each rod. Although these methods demonstrate considerable efficacy in resolving the issue of achieving uniform temperature distribution, they necessitate the use of individual controllers for each heating rod, thereby escalating manufacturing expenses. The prevailing approach of individually controlling each heating rod in sintering molds lacks consideration for cost factors. Simultaneously optimizing the geometric parameters and control methods of the mold can meet equipment design requirements at minimum cost, leading to significant economic benefits. However, there is currently a scarcity of design methods that comprehensively address both performance and economic considerations.

In the present work, an optimization design method that integrated the RSM model with the SQP algorithm was proposed, aimed at elevating temperature uniformity and minimizing control system costs for sintering mold. Firstly, the simplified numerical model containing four pivotal design parameters was established. Then, we established the RSM models for critical temperature-related criteria through the application of Design of Experiments (DoE). The robustness and reliability of these models were comprehensively evaluated through variance analysis, residual analysis, and generalization capability validation. Subsequently, we developed a nonlinear constrained optimization model based on the validated RSM models and employed the SQP algorithm to search for optimal design parameters in the design space. The effectiveness of the proposed RSM-SQP method was substantiated through the validation of optimal design parameters on the complete numerical model, affirming its predictive accuracy and reliability. Finally, parameter sensitivity analysis was employed to assess the extent of parameters' impact on temperature uniformity. Three-dimensional response surface diagrams were constructed to visualize the effect of design parameters on the temperature uniformity.

## 2 Optimization of sintering mold based on surrogate model and SQP algorithm

### 2.1 Numerical modelling of sintering mold

The primary structure of the sintering mold is depicted in Fig. 1(a)-(b). This mold incorporates a heating system consisting of multiple sintering cavities positioned on the surface and 11 heating rods. To enhance cooling efficiency in industrial applications, the heating system is designed with S-shaped water-cooling channels [20,21]. The layout of heating rods and their power density configuration are critical in achieving uniform temperature distribution. Fig. 1(b) depicts two geometric parameters, denoted as *L* and *H*, and two power density parameters labeled as *p*_1_ and *p*_2_. Their specific meanings and range are elucidated in Table 1. Minimizing the number of temperature control units is essential to optimize equipment manufacturing costs. Applying identical power to all heating rods would result in lower temperatures on both sides of the mold, disrupting temperature uniformity. To minimize manufacturing costs and meet the temperature uniformity requirements, the power of the heating rods is controlled in two groups: the outermost two heating rods on both sides constitute one group, while the remaining heating rods form the other group.

**Fig. 1:** (a) Overall structure of mold. (b) the heating system. (c) a quarter geometric model of lower mold.

**Table 1:** Design variables and range.

Design variable	Meaning	Range
*L* (mm)	Distance between two adjacent heating rods	27–30
*H* (mm)	Distance from the heating rod to the cavity surface	8–12
*p*_1_ (W/cm^2^)	Power density of the outermost heating rods	3.5–5
*p*_2_ (W/cm^2^)	Power density of the inside heating rods	2–3.5

The numerical analysis is constructed to assess the temperature uniformity. This study analyzes a quarter model to optimize computational resources, as shown in Fig. 1(c). The minor features, such as threads, holes, and cooling channel are omitted, and the sintering area has been meshed more finely. The main part of the heating system is made of H13 steel, while the remaining components are fabricated using heat insulation panels. The thermophysical properties of components are presented in Table 2. The thermal properties of these materials are regarded as constants during the sintering process. The surfaces in contact with the air are assumed to cool by still air with an equivalent convection coefficient set as 10 W m^−2^ K^−1^, and heat radiation is neglected. The ambient temperature is maintained at 22 °C. Heating flux is applied to the inner walls of the heating rods' mounting holes. In this work, the rate of temperature increase is set at 10 °C/min, as shown in Fig. 1(a). Therefore, the maximum temperature difference observed on the cavity surfaces at the end of the temperature rise phase is selected as the metric for assessing temperature uniformity.

**Table 2:** Material properties.

Material	Density (kg/m^3^)	Specific heat (J/(kg·K))	Thermal conductivity (W/(m·K))
Mold steel H13	7850	460	29
Insulation board	2400	1000	0.21

### 2.2 Optimization method based on RSM model and SQP algorithm

The flowchart of the optimization design process for the heating system of a sintering mold is presented in Fig. 2. The initial phase of the optimization process involves the construction and validation of the surrogate model. The preceding analysis reveals that the four parameters outlined in Table 1 possess the potential to exert a crucial influence on temperature uniformity. The RSM model is accurate enough to characterize the relationship between these four parameters and response. To ensure the cavity surface temperature and temperature uniformity, it is essential to develop RSM models for the maximum temperature difference (Δ*T*), maximum temperature (*T*_max_), and minimum temperature (*T*_min_), respectively. The second-order polynomial regression equation is the most utilized across diverse applications. It can be expressed as follows:

(1) $$y=\beta_{0}+\sum_{i=1}^{n}\beta_{i}x_{i}+\sum_{i=1}^{n-1}\sum_{j>i}^{n}\beta_{ij}x_{i}x_{j}+\sum_{i=1}^{n}\beta_{ii}x_{i}^{2}+\varepsilon$$

**Fig. 2:** Flow chart of optimization design for heating system of sintering mold.

here, *y* represents the objective functions; *x*_*i*_ denotes the design variables, and *n* is the number of design variables. The coefficients ***β***_0_, ***β***_*i*_, ***β***_*ij*_, and ***β***_*ii*_ correspond to the constant, linear, interactive, and quadratic terms, respectively. And *ε* means the statistical error.

A sufficient number of numerical samples are required to fit the RSM models. The central composite design (CCD), involving five levels for each design variable, was utilized to generate the necessary experiment points. ANSYS conducted numerical simulations sequentially to obtain values of Δ*T*, *T*_min_, and *T*_max_ corresponding to the sampled parameter sets. Consequently, the second-order RSM models can be developed by fitting the corresponding data.

During the construction of the RSM models, analysis of variance (ANOVA) played a pivotal role in simplifying the model and confirming its reliability [15,22] The *P*-value is an essential indicator for determining the statistical significance of each model term. A low *P*-value indicates a substantial influence on the response variable. The significance level, commonly denoted as α, is typically set at 0.05 or 0.01. In this article, we adopted a significance threshold of 0.05. Minor quadratic terms exhibiting a *P*-value exceeding the 0.05 threshold were excluded from the analysis to simplify the models. Subsequently, the response surface regression equations were recalculated, omitting these less significant quadratic terms. Additionally, the *F*-value [23], a crucial statistic in ANOVA, was calculated to ascertain the model's reliability. An elevated *F*-value suggests high reliability in the model's predictive capabilities.

It is crucial to validate the prediction accuracy of the developed models before proceeding to the optimization in the subsequent step. Nevertheless, it is not enough to evaluate the reliability of the models only through ANOVA. In our study, a residual analysis was conducted to assess the reliability of the RSM models by examining error normality. Furthermore, three additional validated simulations were performed using random combinations of design parameters within the design space to evaluate the developed models' generalization capability. These validations ensure a comprehensive evaluation of the models’ applicability and robustness.

The objective of the optimization is to achieve the target sintering temperature of 250 °C, with an allowable temperature deviation of ±5 °C. Therefore, the maximum temperature difference of cavity surface Δ*T* should be employed as the objective function. *T*_min_ and *T*_max_ serve as constraints to ensure the temperature remains within the specified operating range. The optimal design of the sintering mold heating system poses a nonlinear constrained optimization problem. The optimization model can be expressed as:

Find *D*, *H*, *p*_1_, *p*_2_

Minimize Δ*T* (*D*, *H*, *p*_1_, *p*_2_)

Subject to $T_{\min}\left(D,H,{\;p}_{1},p_{2}\right)\geq 245,T_{\max}\left(D,H,{\;p}_{1},p_{2}\right)\leq 255\text{,}$.

27≤L≤30,8≤H≤12

(2) $${3.5\leq p}_{1}\leq 5,{2\leq p}_{2}\leq 3.5$$

The SQP algorithm is widely used to solve nonlinear constrained optimization problems because of its super-linear convergence characteristics [19,24,25]. Consequently, this algorithm was adopted to solve the optimization model in Eq. (2). The central concept of the SQP algorithm is transforming the original nonlinear constrained optimization problem into a series of quadratic programming subproblems, formally represented as Eq. (3).

Minimize $\nabla {f\left(x\right)}^{T}d_{k}+\frac{1}{2}d_{k}^{T}B_{k}$.

Subject to $g_{i}\left(x\right)+\nabla {g_{i}\left(x\right)d}_{k}\leq 0$.

(3) $$h_{j}\left(x\right)+\nabla {h_{j}\left(x\right)d}_{k}=0$$

where *f* (*x*) is the objection function, *x* is the design variable, *g*_*i*_ (*x*) and *h*_*j*_ (*x*) are inequality and equality constraint functions. *d*_*k*_ is the iterative search direction and *B*_*k*_ is the Hessian matrix of the Lagrange function.

After determining the optimal design parameters through the RSM-SQP method, validating their reliability is essential. We designed a complete sintering mold based on the optimal design parameters and conducted finite element analysis to ensure our design approach's robustness and applicability.

## 3 Results and discussion

### 3.1 RSM models and validation

Considering the accuracy and complexity of the model, 25 experiment points were generated in design space by the statistical software Minitab using the CCD method. The sampled parameter sets and the corresponding finite element analysis results of Δ*T*, *T*_min_, and *T*_max_ are shown in Table 3. Through fitting the available data, we derived initial response surface models for three temperature-related criteria. The *P*-value of each model term in response surface regression equations are shown in Fig. 3. Since the model terms with *P*-value less than 0.05 are considered significant, according to the fitting results, the quadratic terms with *P*-values greater than 0.05 were not significant, and these quadratic terms were eliminated from the final RSM models. Lastly, the following second-order regression equations without minor quadratic terms were attained by fitting the data again, as shown in Ep. (4)–(6). The *F*-values of Δ*T*, *T*_min_, and *T*_max_ are 49.03, 820.25, and 1567.1, respectively, which implies the models are significant.

**Table 3:** CCD experimental design and numerical results.

No.	Design variable				Response		
	*D* (mm)	*H* (mm)	*p*_1_ (W/cm^2^)	*p*_2_ (W/cm^2^)	*T*_min_ (°C)	*T*_max_ (°C)	△*T*_max_ (°C)
1	25.5	10	4.25	2.75	201.17	249.23	48.06
2	27	12	5	2	191.12	200.58	9.46
3	27	12	3.5	3.5	227.94	287.26	59.32
4	27	12	5	3.5	254.98	297.05	42.07
5	27	8	5	3.5	256.77	301.19	44.42
6	27	8	3.5	3.5	229.05	291.41	62.36
7	27	12	3.5	2	166.72	183.37	16.65
8	27	8	5	2	192.10	205.16	13.06
9	27	8	3.5	2	168.03	185.73	17.70
10	28.5	10	4.25	1.25	131.45	158.8	27.35
11	28.5	10	4.25	2.75	221.88	234.54	12.66
12	28.5	6	4.25	2.75	224.97	239.95	14.98
13	28.5	10	5.75	2.75	240.20	253.22	13.02
14	28.5	14	4.25	2.75	218.94	232.18	13.24
15	28.5	10	4.25	4.25	285.86	336.14	50.28
16	28.5	10	2.75	2.75	192.73	225.26	32.53
17	30	8	5	2	180.98	211.40	30.42
18	30	8	3.5	3.5	247.59	275.46	27.87
19	30	12	3.5	3.5	245.21	271.43	26.22
20	30	12	5	2	180.26	208.25	27.99
21	30	8	5	3.5	275.54	284.33	8.79
22	30	8	3.5	2	171.96	181.47	9.51
23	30	12	5	3.5	273.82	280.30	6.48
24	30	12	3.5	2	171.23	179.19	7.96
25	31.5	10	4.25	2.75	218.49	231.98	13.49

**Fig. 3:** (a) *P*-value of Δ*T* model terms. (b) *P*-value of *T*_min_ model terms. (c) *P*-value of *T*_max_ model terms.(4)$\Delta T=1396-102.8L-0.447H-86.4p_{1}+247p_{2}+1.931L^{2}+4.17p_{1}^{2}+11.3p_{2}^{2}+2.730Lp_{1}-8.768Lp_{2}-11.46p_{1}p_{2}$(5)$T_{\min}=-960+71.1L‐0.475H+66.5p_{1}-77.2p_{2}-1.316L^{2}-2.316p_{1}^{2}-5.787p_{2}^{2}-1.590Lp_{1}+4.831Lp_{2}+4.978p_{1}p_{2}$(6)$T_{\max}=436-31.68L-0.922H-19.9p_{1}+169.9p_{2}+0.615L^{2}+1.852p_{1}^{2}+5.510p_{2}^{2}+1.140Lp_{1}-3.937Lp_{2}-6.480p_{1}p_{2}$

The residual analysis results of the RSM models are shown in Fig. 4. We can see that the residual error of Δ*T*, *T*_min_, and *T*_max_ align closely with a straight line, confirming that the error follows a normal distribution. This affirms that the mathematical models have been appropriately fitted using the least squares regression technique. To assess the generalization capability of the previously acquired models, three distinct sets of parameter combinations were randomly generated within the design space. Special care was taken to ensure that these parameter sets differed as much as possible from the parameter sets used in 25 experiment points. The three sets of parameters and their corresponding finite element analysis results are shown in Fig. 5. The predicted error (δ), representing the variance between the predicted value of the RSM model and the simulation result from finite element analysis, serves as a critical criteria of the model's generalization capability. From Fig. 5 we can see that among the three parameter combinations, all the absolute errors of Δ*T*, *T*_min_ and *T*_max_ are less than 2 °C, indicating that the developed RSM models can provide highly accurate predictions within the design space.

**Fig. 4:** The normal probability distribution diagram of the standardized residual. (a) Δ*T*. (b) *T*_min_. (c) *T*_max_.

**Fig. 5:** Predicted errors of RSM models for three random parameters combinations.

Following a comprehensive examination involving variance analysis, residual analysis, and verification of generalization capability, the reliability of RSM models has been firmly affirmed. As a result, the reliance on finite element simulation to obtain temperature-related criteria for any parameter combination within design space is now rendered unnecessary. Accurate values can be directly derived through the application of the response surface models.

### 3.2 Optimal design based on RSM models and SQP algorithm

The optimization iteration process of the RSM-SQP method is shown in Fig. 6(a). As can be seen, the fitness value gradually decreases with the iteration number increasing. After 9 iterative calculations, the optimization process is terminated, and then the optimal parameters are obtained. The optimal parameters and their corresponding maximum temperature difference in the sintering area are illustrated in Fig. 6(b). With the optimal parameters, the maximum temperature within the sintering area is 254.83 °C, and the minimum temperature is 246.59 °C, resulting in a maximum temperature difference of 7.38 °C. Notably, both the maximum and minimum temperatures fall within the range of 245–255 °C, indicating an elevated level of temperature uniformity in the sintering area. To ascertain the superiority of the RSM-SQP method, we compared the maximum temperature difference in the sintering area obtained under optimal parameters with that under the initial design parameters. The initial design parameters, generated by random combinations within the design space, serve as the starting point for the RSM-SQP method. The initial parameters and the corresponding three temperature-related criteria results are shown in Fig. 6(b). Both the maximum and minimum temperatures in the sintering area significantly surpass the design specifications. Moreover, the temperature uniformity was extremely poor, with the maximum temperature difference exceeding 30 °C. Through optimization, the temperature difference is reduced by 75.8 %. The RSM-SQP method shows excellent performance in improving the temperature uniformity of the sintering mold.

**Fig. 6:** (a) Optimization iteration process of SQP algorithm. (b) design parameters and predicted values before and after optimization.

We designed the complete sintering mold using the optimal parameters obtained from the simplified quarter model and performed finite element simulations. The temperature distribution of the complete sintering mold is shown in Fig. 7(a). Due to the enhanced heat dissipation at the periphery of the heating plate compared to its central area, the temperature at the plate's middle surpasses that of its surroundings, with both ends experiencing lower temperatures. Within the optimal parameters, the outermost heating rods display a power density of 4.76 W/cm^3^, while the inner heating rods have a power density of 3.08 W/cm^3^. Notably, this significant difference in power density between the outermost and inner heating rods effectively compensates for the heightened heat emission from the outermost section, ensuring a more even temperature distribution. The temperature distribution in the sintering area is shown in Fig. 7(b). The cavity surface exhibits a temperature range from 248.43 °C to 252.46 °C, with a maximum temperature difference of 4.03 °C. These results demonstrate exceptional temperature uniformity throughout the entire cavity surface, further confirming the robustness and reliability of the RSM-SQP algorithm proposed in this study for optimizing the mold heating system.

**Fig. 7:** Optimal parameters simulation results. (a) overall temperature distribution. (b) temperature distribution of cavity surface.

### 3.3 Parameter analysis

#### 3.3.1 Parameter sensitivity analysis

Parameter sensitivity analysis is commonly employed to assess the extent of parameters' impact on the response. To explore the influence of each design parameter on temperature uniformity, we conducted a detailed quantitative assessment of parameter sensitivity, utilizing the standardized effect as a crucial analytical approach. All independent variables are standardized, ensuring they can be compared within the same measurement scale. A regression analysis is conducted using the standardized independent variables to derive the standardized regression equation. The absolute value of T-statistic is defined as the standardized effect. The T statistic is calculated by dividing the standardized regression coefficient for each term by the corresponding standard error. A higher standardized effect value indicates a more substantial impact of the factor on the response variable.

The regression coefficients and standard errors of the standardized regression equation for Δ*T* are shown in Table 4. The standardized effects of each factor and their interactions on Δ*T* are illustrated in Fig. 8. It is evident that the distance between two adjacent heating rods (*L*) and the power density of the inside heating rods (*p*_2_) exert the most significant influence on the cavity surface temperature difference, with their effects being nearly equivalent. The next most influential design parameter is the power density of the outermost heating rods (*p*_1_), while the distance between the heating rod and the cavity surface (*H*) has the least impact on temperature uniformity. Furthermore, the interaction between *L* and *p*_2_ exhibits a notable impact on temperature uniformity. Simultaneously, the interaction between *p*_1_ and *p*_2_ also exerts a considerable impact on temperature uniformity. Therefore, particular emphasis should be given to the *L*, *p*_1_ and *p*_2_ when designing the heating system of sintering mold.

**Table 4:** Regression coefficient and standard error of standardized regression equation.

Term	constant	*L*	*H*	*p*_1_	*p*_2_	*L-L*	*p*_1_- *p*_1_	*p*_2_- *p*_2_	*L*- *p*_1_	*L*- *p*_2_	*p*_1_- *p*_2_
Regression coefficient	12.86	−7.873	−0.894	−3.947	7.943	4.345	2.345	6.355	3.071	−9.864	−6.445
Standard error of coefficient	1.26	0.789	0.789	0.789	0.789	0.718	0.718	0.718	0.966	0.966	0.966

**Fig. 8:** (a) Standardized effects of single factors. (b) standardized effects of coupling factors.

#### 3.3.2 The effect of main design parameters on temperature uniformity

To visualize the effect of design parameters on temperature uniformity, three-dimensional response surface diagrams can be used to describe the extracted mathematical models [8,26,27]. Through the previous parameter sensitivity analysis, we know that *L*, *p*_1_, *p*_2_, and their interactions have a significant impact on temperature uniformity. Hence, we generated three-dimensional response surface diagrams of Δ*T* with respect to these three design parameters, as shown in Fig. 9.

**Fig. 9:** Response surface contour of Δ*T*. (a) the interaction between *L* and *p*_1_. (b) the interaction between *L* and *p*_2_. (c) the interaction between *p*_1_ and *p*_2_.

The effect of the distance between two adjacent heating rods and the power density of the outermost heating rods is shown in Fig. 9(a). Additionally, Fig. 9(b) elucidates the relationship between the distance between two adjacent heating rods and the power density of the inside heating rods. It is evident that Δ*T* exhibits a decrease with an increase in the distance between adjacent heating rods. Specifically, a considerable distance between two adjacent heating rods results in a relatively minor influence of the heating rods power density on temperature uniformity. Conversely, a reduced distance accentuates the impact of heating rods power density on temperature uniformity. Fig. 9(c) explores the interaction between the power density of the outermost heating rods and that of the inner heating rods. Notably, when the power density of the inner heating rods is set to a smaller value, the effect of the outermost heating rods power density on temperature uniformity is diminished. In conclusion, optimal temperature uniformity is achieved by adopting a larger distance between heating rods and configuring the power density of the heating rods to a relatively modest level.

## 4 Conclusion

In this study, we introduced an optimization approach that combines RSM surrogate models with the SQP algorithm to optimize the geometric parameters and heating power configuration of a heating system for sintering mold. This methodology concurrently considers both temperature uniformity and manufacturing cost in the optimization process. According to the results obtained in our research, the following conclusions can be drawn.

A strategic approach was employed to achieve a reduction in manufacturing costs alongside the optimization of geometric parameters. We classified the 11 heating rods into two distinct control groups: the first group comprised the outer two rods, while the remaining nine constituted the second group. The RSM models for critical temperature criteria were developed, including Δ*T*, *T*_min_, and *T*_max_. The reliability of these RSM models was systematically affirmed through variance analysis, residual analysis, and generalization capability validation. The response surface models demonstrate remarkable predictive accuracy within the design space.

A nonlinear constrained optimization model was established based on the RSM models, and the optimal parameters were obtained using the SQP algorithm. The RSM-SQP method exhibited rapid convergence, achieving optimal design parameters after only 9 iterations. These optimal design parameters led to a remarkable 75.8 % reduction in predicted maximum temperature difference compared to the initial design parameters. A complete sintering mold was designed based on optimal parameters, and the reliability of the optimal parameters was verified through FEM simulation. Significantly, the maximum temperature difference observed on the cavity surface was a mere 4.03 °C, affirming the exceptional temperature uniformity across the cavity surface.

The parameter sensitivity analysis based on standardized effects was conducted to assess the influence of design parameters on temperature uniformity. The results shown that the distance between two adjacent heating rods and the power density of the inside heating rods exert the most significant influence on the temperature difference. The distance from the centre of the heating rod to the cavity surface has the weakest impact. Furthermore, the interaction between the distance between two adjacent heating rods and the power density of the inside heating rods exhibits a notable impact. Additionally, the interaction between the power density of both inner and outermost heating rods exerts a substantial impact on temperature uniformity. Therefore, particular emphasis should be given to the *L*, *p*_1_ and *p*_2_ when designing the heating system of sintering mold. By analyse the three-dimensional response surface diagrams of Δ*T* with respect to these three design parameters, the optimal temperature uniformity can be attained by increasing the distance between heating rods and adjusting the power density of the heating rods to a relatively moderate level.

This work introduces a practical approach to optimize the heating systems for sintering molds, offering promising prospects for application across diverse industrial mold optimization.

## Funding statement

This work was supported by the Natural Science Foundation of Shanghai, China [21ZR1424100], 10.13039/501100006683XJTLU Research Development Fund [RDF-17-02-44, RDF-SP-122] and Industrial Research & Development Fund [RP0029].

## Data availability statement

Data included in article/supp. material/referenced in article.

## Additional information

No additional information is available for this paper.

## CRediT authorship contribution statement

**Sanli Liu:** Writing – original draft, Methodology. **Min Chen:** Writing – review & editing. **Nan Zhu:** Validation. **Zhouyi Xiang:** Software. **Songhua Huang:** Software. **Shunqi Zhang:** Resources.

## Declaration of competing interest

The authors declare the following financial interests/personal relationships which may be considered as potential competing interests:Shunqi Zhang reports financial support was provided by Natural Science Foundation of Shanghai. Min Chen reports financial support was provided by Xi'an Jiaotong-Liverpool University. If there are other authors, they declare that they have no known competing financial interests or personal relationships that could have appeared to influence the work reported in this paper.
